This article has been retracted.

# Construction of the Maximum Oxygen Intake Regression Equations for Exercise Training on Respiration and Heart Rate

**DOI:** 10.1155/2022/6281199

**Published:** 2022-03-07

**Authors:** Kai Kang

**Affiliations:** North China University of Water Resources and Electric Power, Zhengzhou 45000, Henan, China

## Abstract

To explore the correlation between the maximum percentage heart rate and the maximum percentage oxygen intake, provide an evaluation basis for heart rate for the assessment of exercise load intensity. Four boys and 4 girls were randomly selected, aged 26.25 ± 2.12 years old with good health, good cardiopulmonary function, no other medical history, and irregular physical training history. The subject measured the first 30 min of rest at 25°C at room temperature, kept awake and static, and the heart rate was measured as the quiet heart rate in the state. Prepredicted maximum heart rate and health index were determined according to the Polar s810 heart rate table instructions. Prepredicted maximum heart rate and health index were measured three consecutive times and reliability analysis was performed on three measurements. The regression equations were established by a stepwise method with data represented that all metrics were tested for normality for fitness index and maximum oxygen intake compared using a paired *t* test with a significance level of *P* < 0.05. The results showed that the highest value of VO_2max_ motor cardiopulmonary test was 47.83 ml/(kg·min), the lowest was 35.06 ml/(kg·min), the two-step test was 44.50 ml/(kg·min), and the lowest was 32.89 ml/(kg min).With a positive correlation between the postexercise heart rate and the maximum oxygen intake, the maximum oxygen intake value can be indirectly inferred using the heart rate after the exercise and the work completed by the exercise. The results measured by two-step test have some accuracy and can be used to speculate the maximum oxygen intake in the ordinary young population. The polar heart rate meter allows subjects to indirectly measure the maximum oxygen intake in silence, requiring less equipment and being easy to operate. The indirect measurement of the maximum oxygen intake can be used for the monitoring of competitive sports and national fitness.

## 1. Introduction

The maximum oxygen intake is the amount of oxygen that can be taken per unit time during the cardiopulmonary function and the capacity of muscle to reach the extreme oxygen in a large amount of muscle participation, which is one of the commonly used important indicators to evaluate the human body's aerobic endurance [1]. Maximum oxygen intake was measured by both direct and indirect methods. The direct method obtains by increasing load movement to measure the oxygen intake when the body reaches the maximum limit level of oxygen capacity [2]. Although the proposed method can directly obtain the real maximum oxygen intake value, the measurement method is complex, high condition demand, long time consuming, large increasing motion load, and difficult to subjects and cannot be used for large sample measurement, so it is usually used with simple indirect method [3]. Indirect method includes a variety of methods, and the more commonly used method is the subpolar step motion test. By measuring the exercise heart rate of the human body, the maximum oxygen intake is calculated by the regression formula.

The maximum oxygen intake is the oxygen content absorbed and utilized by the body in a unit of time under the condition of cardiopulmonary function and systemic organs and full mobilization of the system. It can be divided into absolute maximum oxygen intake and relative maximum oxygen intake. Absolute value units are expressed as L/min; relative value units are expressed as mL/(kg∗min). The factors affecting the maximum oxygen intake mainly determine the oxygen transport capacity and the oxygen capture capacity of peripheral tissues [4]. Maximum oxygen intake is an important indicator to evaluate the human aerobic work capacity. Before the start of the rehabilitation training and during the training process, it is necessary to understand the cardiopulmonary oxygen supply capacity and evaluate the cardiopulmonary endurance in order to guide the exercise prescription and assess the efficacy. There are many indicators for the evaluation of cardiopulmonary function. At present, the maximum oxygen intake (VO_2max_) and anaerobic threshold (VT) are commonly used to reflect the aerobic endurance level. Sports physiologists at home and abroad agree that the best index to evaluate the cardiopulmonary mechanical capability is the maximum oxygen intake (VO_2max_). VO_2max_ refers to the maximum oxygen amount consumed and supplied by tissue cells when the body reaches the maximum power amount, which is an important indicator reflecting the body's aerobic exercise ability. VO_2max_ was determined by both direct and indirect methods [5]. The effect of the high quality of circulating circulation on vascular function and heart and lung function in sedentary humans was investigated by Chidnok et al. Methods: twenty-two female participants were divided into two groups, including the HIIT group receiving no intervention and the control group. Each participant interviewed, collected, and recorded their history and medical parameters including cardiac ankle vascular index (CAVI), flow-mediated dilation (FMD), and maximum oxygen consumption (VO2MAX) which were included as baseline predictors. The intervention was a circular HIIT lasting for 6 weeks with three courses per week. During each session, participants completed a set protocol consisting of 1 min on the cyclic force meter, with a maximum heart rate cycle of 80–85% and then rested. The sequence was repeated in total of 5 times. Results: after 6 weeks of the intervention, the results indicated that the HIIT group was in CAVI (6.39 ± 0.76 vs. 5.91 ± 0.58), FMD (9.26 ± 6.5 and 14.01 ± 4.3%), and vo_2max_ (20.10 ± 4.31 vs. 24.34 ± 5.71 ml/kg/min) values as compared to the predictive trials (*P* < 0.05). In addition, the increased endothelial function of HIIT is measured by FMD compared to controls (14.01 ± 4.3 versus 9.15 ± 4.16%, *P* < 0.05). Conclusions: six weeks of HIIT improved vascular and cardiopulmonary function in poor people and demonstrate the benefits as a stable exercise strategy [6].

Based on the basis of this study, the two-step test and the motor cardiopulmonary function test were used to analyze whether the difference between the two was statistically significant and find out the speculative method of the maximum oxygen intake of ordinary young population. Subjects measured the quiet heart rate, predicted maximum heart rate, and health index using fitness tests from the Polar s810 heart rate table to speculate on maximum oxygen intake. Subjects in this experiment did not need to test against a specific exercise procedure and could directly derive the maximum oxygen intake in a quiet state.

## 2. Research Method

### 2.1. Research Object

4 boys and 4 girls were randomly selected aged 26.25 ± 2.12 years old with good health, good cardiopulmonary function, no other medical history, irregular physical training, and voluntary participation in this trial.

### 2.2. Methods

The quiet heart rate, predicted maximum heart rate, and health index were tested by polar S810 heart rate meter. The subjects rested in a quiet environment (room temperature 25°C) for 30 minutes and remained awake and static before measurement. the determination of heart rate is quiet heart rate. Prepredicted maximum heart rate and health index were determined according to the Polar s810 heart rate table instructions. Prepredicted maximum heart rate and health index were measured three consecutive times and reliability analysis was performed on three measurements.

Determination of the maximum oxygen intake: the subject performed the increasing load exercise on the MONARK821 power bicycle, and the maximum oxygen intake was directly measured using the American type PHYSIO-DYNEMAX-1 gas analyzer. The maintenance speed is 60r/min, the power load starts at 60W, and the power increases by 30 W, every 3 points until the subject reaches the determination standard state P2, at maximum oxygen intake, i. e., the oxygen intake difference is less than 5% or 150 mI/min or 2 mL/(kg∗min). ② Breathing quotient >1.10; heart rate >180 times/min. A decrease in oxygen intake occurred as the ③ continued to exercise.

#### 2.2.1. Direct Assay

The maximum oxygen intake was automatically calculated by using the automatic cardiopulmonary function analyzer. Use instrument: power activity plate and cardiopulmonary function automatic analyzer. Subjects wore a breathing mask, exhaled gas was connected to a gas analyzer, and then performed incremental load movement on a power active plate or on a power bicycle, which automatically recorded heart rate, ventilation, and oxygen intake every minute. The oxygen intake increases with the increasing load. This amount of the oxygen intake was the maximum oxygen intake when the subject had >1.2 (the ratio of CO_2_ discharge to O_2_ intake), the oxygen intake no longer increased (or <2 ml/min), or the subject reached maximum fatigue and could longer continue exercise.

#### 2.2.2. Indirect Determination Method

Two-step test method: the test instrument is the instrument stipulated by the national physical health test standard. Subjects followed the beat up and down the steps and exercise lasted 3 min; subjects followed the rhythm up and down the steps (18 cm two steps) at the frequency of 134/min, exercise standing 1 min; each subject wore a polar table, recording the heart rate throughout the trial. The maximum oxygen intake is as follows:

(1) $$\begin{array}{c} {\text{VO}}_{2\max}={\text{HR}}_{\max}\times \frac{{\text{Vo}}_{2}}{\text{HR}}, \end{array}$$

HR_max_ (male) = 220-age, HR_max_ (female) = 210-age; VO_2_ is the exercise intensity; movement intensity is 28.9 ml/(kg·min) at 134 times/min frequency; heart rate × 6 at 10s after the end of the HR = exercise.

### 2.3. Data Analysis and Methods

Statistical analysis: data statistical analysis was completed using SPSS11.5 statistical software, and the data map was generated by version sigmaplotforwindows8.0. Data are expressed, all metrics were tested for normality, and the health index and maximum oxygen intake were compared using a paired *t* test with a significance level of *P* < 0.05. The ratio of health index and body mass was then analyzed by Pearson correlation with the maximum oxygen intake, and then the regression equation was established by stepwise regression.

## 3. Result Analysis

The highest value of the VO_2max_ motor cardiorespiratory test was 47.83 ml/(kg min), the minimum was 35.06 ml/(kg min), the two-step test was 44.50 ml/(kg min), and the minimum was 32.89 ml/(kg min) (see Table 1). Correlation analysis of heart rate and VO_2max_ values in group 2 subjects is shown in Figures 1 and 2. Heart rate was significantly associated with VO_2max_ after a two-step trial and motor heart and lung function trial (*P* < 0.05). The results of two-step and motor cardiopulmonary function test met the law with normal distribution. *t* tests of two paired samples were performed on two sets of VO_2max_ data. The results showed that the two-step test and the VO_2max_ values were not significantly different (*P* < 0.05).

The subjects' quiet heart rate and predicted maximum heart rate were 76.314 ± 0.3/min and 193.2 ± 3.2/min, respectively, and the ratio of the predicted maximum heart rate to body weight was 2.8 ± 0.3, the ratio of health index to body weight was 0.6 ± 0.1, and the difference between maximum oxygen intake (45.9 ± 5.7 L/min) and health index was significant *P* < 0.05. Test results for predicted maximum heart rate and health index reliability for 16 subjects with 3 predictions were (181.6 + 3.2), (181.9 soil 3.2), (182.2 ± 3.1)/min; subjects' predicted maximum heart rate was 0.9965, *P*=0.0178; 3 test values were (41.0 + 7.4), (41.5 + 7.3), and (41.8 ± 7.3) L/min; health index was 0.9958, *P*=0.043. Three test values indicate high reliability and good reproducibility for the predicted maximum heart rate and health index.

Scatter plot of subjects' predicted maximum heart rate body mass ratio to maximum oxygen intake is shown in Figure 3.

As shown in Figure 3, the predicted correlation coefficient of the maximum heart rate mass and the maximum amount of oxygen content is 0.541, which is highly correlated, and the regression equation can be established by test *P* < 0.05. With the ratio of the maximum heart rate and the quality of the body, the regression equation established by the gradual regression of the gradual regression is $\hat{y}=11.6x+13.8$; the standard estimation error = 5.0, *P*=O.11.

## 4. Discussion

1. According to the results of this test, there is a correlation between heart rate and VO_2max_ value after exercise. In the two-step trial, heart rate was more associated with VO_2max_ than in the motor cardiopulmonary function trial. The reason is that heart rate not only reflects the frequency of heart beating but also reliably reflects the cardiovascular function of the human body, through which it can more accurately understand the immediate response or chronic adaptation to motor stimulation. Therefore, the subject's VO_2max_ can be calculated indirectly by using the measured postexercise heart rate.
2. The VO_2max_ motor cardiorespiratory function test method synchronously evaluates the individual function of multiple organ systems in the motor state, including the respiratory system, cardiovascular system, hematopoietic system, neuropsychological system, and skeletal muscle system, by measuring the gas exchange in the respiratory tract. The VO_2max_ results measured by two-step test and motor cardiopulmonary function test were not significantly different (*P* > 0.05), and the two-step test had certain accuracy and feasibility.
3. In the two-step trial, only two-step and heart rate meter were used, which cost less relative to the platform and cardiopulmonary analyzer in the exercise cardiopulmonary function test. The trial process takes 3∼5 min, is short time consuming, and physical fitness tests are widely adopted by domestic universities, while exercise cardiopulmonary tests require research in large research and medical places for [7]. The step test is an effective exercise load evaluation test of the cardiovascular system, but it can only make good and bad general judgment on the cardiovascular function level, without accurate judgment; the step test has good measurement reliability; the step test score is more sensitive to the exercise effect than the maximum oxygen consumption.
4. Clinical significance: exercise cardiopulmonary function test is more suitable for groups with cardiovascular disease to test. It is widely used in other diseases, such as chronic heart failure. Respiratory diseases are mainly used in the pathological research and efficacy evaluation of COPD, as well as some other lung diseases, such as sleep apnea syndrome and asthma. The exercise cardiopulmonary function test is highly safe and more suitable for groups with cardiovascular disease. Compared with the exercise cardiopulmonary function test, the obvious advantage of the step test is that it can test a large number of people at the same time, and the tester does not need special training, and the test instruments are cheap. Therefore, in general, the two-step test method is simpler than the exercise cardiopulmonary function test method.

Maximum oxygen intake is the amount of oxygen actual and consumed per minute at the maximum functional levels of breathing, circulation, and the skeletal system. It is a comprehensive measure of respiratory circulation and muscle system. It can reflect the body's maximum aerobic work ability and reflect the muscle transport oxygen and oxygen (including heart displacement, hemoglobin, and capillary density) and muscle oxygen (including mitochondria and enzymatic activity). In the method of directly testing the maximum oxygen intake, the more the muscles involved in exercise, the greater the oxygen intake; the running with slope is larger than the maximum oxygen intake without slope, and the running is the maximum oxygen intake than riding a bicycle. The direct determination of the maximum oxygen intake using a protocol was extremely reproducible, with a coefficient of variation at 2%∼4%. The study shows that the direct measurement of maximum oxygen intake is accurate and reliable, which can comprehensively evaluate cardiopulmonary function and requires precision instrument and equipment [8]. The method is complex, especially with a large load, which is difficult for subjects to accept. Sometimes, danger may occur, so this method should not be popularized. However, the search method is simple and easy to accept, and the indirect speculation maximum oxygen intake method with high accuracy has become the goal of many scholars to explore. The basic idea is to find the physiological indicators related to the maximum oxygen intake and use its correlation to guess the maximum oxygen intake [9]. The more famous indirect measurement is the Swedish exercise physiologists Astrand and Rhyming who proposed the famous Astand–Ryhming physiography; many sports physiologists have proposed different indirect measures, measuring the physiological indicators in different states according to certain exercise procedures to guess the maximum oxygen intake. Chinese scholars have revised some foreign methods according to the characteristics of the Chinese people and put forward their own maximum oxygen intake regression equation [10]. For example, the Chinese scholar Ding Zhenping developed the binary regression prediction equation for the actual measured maximum oxygen intake, which can better reflect the actual maximum oxygen intake. The maximum oxygen intake was also speculated from the power reached when the heart rate was stable at 170 times/min.

## 5. Conclusions

In conclusion, the advantage of this method is that the maximum oxygen intake can be indirectly measured in the case of quiet subjects, requiring less equipment and being easy to operate. After the regression equation is established, it is still needed to be tested in practice and improved in practice. Population, age, gender, and other factors were considered as far as possible. Population, age, gender, and other factors were considered as far as possible. What should be noted in further research is as follows: expand sample size, reduce sampling error, correct debugging and use of test instruments, reduce systematic error, expand the scope of subjects, and assess the aerobic exercise level of rehabilitation training patients.

## Figures and Tables

**Figure 1:** Correlation of HR_max_ in the motor cardiopulmonary function test and VO_2max_.

**Figure 2:** Two-step test HR correlation with VO_2max_.

**Figure 3:** A scatter plot of the maximum heart rate body mass ratio to the maximum oxygen intake is predicted.

**Table 1:** Results of exercise cardiopulmonary test and two-step test.

Method	Pretrial heart rate (secondary/min)	Posttrial heart rate (secondary/min)	Maximal oxygen intake（ml/kg·min)
Exercise heart and lung function test	87.88 ± 10.97	186.00 ± 2.78	39.87 ± 4.75
Two-step test	84.00 ± 4.67	151.50 ± 16.59	37.86 ± 5.12

## Data Availability

The data used to support the findings of this study are available from the author upon request.
